The article "Logistics Path Decision Optimization Method of Fresh Product Export Cold Chain Considering Transportation Risk" was published in 2022. Journal: Comput Intell Neurosci.

# Logistics Path Decision Optimization Method of Fresh Product Export Cold Chain Considering Transportation Risk

**DOI:** 10.1155/2022/8924938

**Published:** 2022-10-07

**Authors:** Lifu Chen, Zhifeng Shen

**Affiliations:** Department of International Economy and Trade, Jiangsu University of Technology, Changzhou 213001, China

## Abstract

The cold chain logistics route of fresh product export is characterized by large quantity and complexity, which is prone to cause transportation risks of different degrees in the process of fresh product export transportation and affects the decision-making effect of the cold chain logistics route. Therefore, in order to improve the ability of cold chain logistics route planning and shorten the transportation time, an optimization method of fresh product export cold chain logistics route decision considering transportation risk was proposed. This paper analyzes the basic characteristics and classification of cold chain logistics by means of risk quantification and uses the K-nearest neighbor algorithm to predict the risk of traffic congestion, so as to shorten the transportation time. Ahp process is used to construct a risk factor judgment matrix and determine the index weight of risk factors, so as to reduce the error of path planning. A genetic algorithm is introduced to construct the optimal decision function of the cold chain logistics route of new product export and realize the optimization of cold chain logistics route decision of fresh product export. Experimental results show that the method presented in this paper can effectively improve the decision-making effect of cold chain logistics route and select the shortest and most smooth transportation path to complete logistics distribution. The decision-making accuracy of the route decision effect is 90%, and the transportation time is 31.45 min, which has certain feasibility and applicability.

## 1. Introduction

Cold chain logistics refers to a systematic engineering of refrigerated and frozen food in the production, storage, transportation, sales, and consumption before all the links are always in the specified low-temperature environment, in order to ensure food quality and reduce food loss. Cold chain logistics has higher requirements, and the corresponding investment in management and capital is also larger than ordinary normal temperature logistics. Therefore, in the process of cold chain logistics transportation of fresh product export, costs must be reduced to ensure actual profits [1]. Domestic transport routes are complex, and transport vehicles often fail to choose the shortest route, which reduces distribution efficiency and improves transport costs [2]. With the rapid development of the economy and the improvement of scientific and technological level, people's demand for food has also changed, among which the demand for cold-chain food has been increasing [3]. However, due to low transportation efficiency, backward facilities, backward technology, and other factors, it takes a long time to transport cold-chain food, resulting in food decay and increasing logistics and transportation costs [4]. As export transportation is affected by many factors, the quality of products in export transportation is affected and more economic costs are wasted [5]. Therefore, it is necessary to carry out a lot of planning and research on the cold chain logistics route of fresh product export. Literature [6] proposed a vehicle route optimization method for multivehicle cold chain logistics of fresh agricultural products. By constructing a multivehicle routing optimization model, the adaptive degree of congestion index is considered on the basis of reducing the overall delivery cost and improving customer satisfaction. The genetic simulated annealing algorithm is used to calculate the total distribution cost of the cold chain logistics path time window to complete the cold chain logistics path planning. The optimization path of this method has some errors and needs to be improved continuously. Literature [7] proposed a method for vehicle routing optimization of cold chain logistics based on the green evaluation. The vehicle path optimization model of cold chain logistics is constructed for the optimization evaluation of total distribution cost. The vehicle evaluation results are considered through the comprehensive method of vehicle evaluation value, so as to obtain the corresponding vehicle path optimization results of cold chain logistics. This method has certain precision, but it ignores the risk interference in transportation and has certain limitations. Literature [8] proposed an optimization method for multitemperature and low-temperature cold chain logistics vehicle distribution route. Considering the interference factors at each stage, the distribution time, distribution cost, and distribution risk of multitemperature cold chain logistics were controlled to optimize the vehicle distribution path of multitemperature cold chain logistics, and the path optimization was realized by the ant colony algorithm. This method can effectively plan the path, but because the ant colony algorithm needs to obtain the optimal value through a large number of calculations, the data results are redundant, which can easily prolong the path optimization time.

In view of the problems in the above methods, this paper proposes an optimization method for cold chain logistics route decision of fresh product export considering transportation risk. Based on the analysis of the basic characteristics and classification of cold chain logistics, a transportation risk factor system of cold chain logistics for new product export considering transportation risks is established based on customs clearance efficiency, vehicle stability, cold chain terminal, traffic congestion, and other factors. The analytic hierarchy process (AHP) is used to obtain the transportation information of the cold chain logistics route of fresh products export, and then the risk factor judgment matrix is constructed to determine the index weight of risk factors. A genetic algorithm is introduced to construct the optimal cold chain logistics route decision function of new product export through encoding, decoding, crossover, and other operations and realize the optimization of cold chain logistics route decision of new product export. The experimental results show that the method proposed in this paper can effectively improve the decision-making effect of the cold chain logistics path. The cold chain logistics path is the shortest, the decision-making accuracy is high, and the transportation time is short, which has certain feasibility and applicability.

## 2. Cold Chain Logistics System

In order to realize the design of the decision-making optimization method of fresh product export cold chain logistics path, this paper first analyzes the risk factors existing in fresh product export cold chain logistics. Cold chain logistics generally refers to the whole process of refrigerated and frozen products from production and transportation to storage or secondary processing in the warehouse, and finally into the hands of consumers through dealers. And the whole process should be strictly controlled in the low-temperature environment. It is a systematic project to ensure product quality, maintain product freshness, and reduce loss through various refrigeration means [9]. Cold chain logistics is a low-temperature logistics process maintained by refrigeration technology and equipment. The general process of cold chain logistics is shown in Figure 1.

Different cold chain products require different storage temperatures. The classification of cold chain products and their characteristics in China are shown in Table 1.

Cold chain logistics is more demanding and complex than traditional logistics systems. In order to ensure that products will not be corroded and damaged, it is necessary to build a complete cold chain system with investment. It takes the low-temperature environment as the core and meets the timeliness requirements of products through reasonable and effective organization and coordination. In order to ensure the low-temperature environment, the cold chain logistics system is generally accompanied by high costs. Therefore, the reasonable classification of cold chain products and the construction of a cold chain logistics system are of great significance to the development of the cold chain industry [10].

## 3. Extraction of Transportation Risk Factors of Cold Chain Logistics Based on Risk Quantification

### 3.1. Establishing the Index System of Cold Chain Logistics Transportation Risk Factors

The risk management of fresh product export cold chain logistics transportation requires to be able to identify the risk, quantify the identified wind direction, and evaluate the risk according to the quantitative results. It also includes the implementation of some risk control methods, decision-making based on risk analysis, and performance evaluation of risk management effect. Risk identification is to collect information such as the possibility of risk occurrence and the number of accidents that have occurred and make probability statistics. There are many methods to identify possible risk factors. Find out the causes of risks according to different links. Generally, experts can identify relevant risks according to their own experience, which is also of great reference significance. In the process of risk identification, many scholars often use a variety of methods together, which can help to identify risk factors as comprehensively as possible. The risk quantification process is mainly based on the analysis of historical basic data, using probability theory and mathematical statistics to quantitatively analyze and describe risk indicators. Reasonable and effective data is the basis of risk quantification because risk quantification must rely on data support. Therefore, this paper analyzes the risk factors of fresh product export cold chain logistics transportation before the decision-making and optimization of the fresh product export cold chain logistics transportation path [11].

In the whole cross-border cold chain logistics transportation process, fresh products are faced with various uncontrollable factors, such as many transportation links, complex transportation process, different transportation subjects involved, and different economic, political, and transportation habits at home and abroad. The risk factor index system of fresh product export cold chain logistics transportation constructed in this paper is shown in Figure 2.

In the transportation process of cross-border cold chain logistics of fresh products, transportation cost, time, mode, transportation volume, and transportation path are usually considered. In addition, due to the differences in storage temperature, storage time, storage time limit, and product value of various agricultural products, more suitable transportation methods and more reasonable transportation paths are adopted for different fresh agricultural products in the whole cross-border logistics transportation process. It can maximize transportation efficiency and reduce transportation risks and costs under the conditions of existing infrastructure.

### 3.2. Extraction of Cold Chain Logistics Transportation Risk Factors

In this paper, considering the customs clearance efficiency, the choice of transportation mode and port will be more objective. Choosing transportation mode and port with higher customs clearance efficiency will make the comprehensive operation efficiency of cross-border cold chain logistics the highest. The customs clearance time per unit cargo volume is used to represent the customs clearance efficiency, but the shorter the time, the higher the customs clearance efficiency [12]. In order to facilitate understanding, the reciprocal is taken in the calculation. At this time, it means that the larger the calculation result is, the higher the customs clearance efficiency is. The calculation formula is

(1) $$\begin{array}{c} A_{in/out}=\frac{N_{i}}{v_{i}}\text{.} \end{array}$$

Here, *A*_*in*/*out*_ represents the customs clearance efficiency of import and export, *v*_*i*_ represents the working time of port *i*, and *N*_*i*_ represents the freight volume exported or imported from port *i*.

In this paper, the stability of vehicles is mainly based on the transportation stability of different vehicles in the cross-border cold chain transportation of fresh agricultural products, so as to ensure the timely and smooth progress of logistics activities. For high-value and perishable products, each route is weighted according to the punctuality rate of each transportation mode in the selection of different transportation modes. The calculation method is shown in the following formula:

(2) $$\begin{array}{c} B_{j}=\frac{c_{j}}{a_{j}}\times 100\%\text{.} \end{array}$$

Here, *B*_*j*_ represents the punctuality rate of transport, *c*_*j*_ is the number of transport *j* arriving on time, and *a*_*j*_ is the total number of transport *j*.

The interruption of the cold chain has a great impact on the quality of fresh products, and the interruption usually occurs at the place of transshipment. Therefore, the probability of interruption is small when the number of loading changes is small. The purpose of selecting this risk index is to replace as little as possible on the basis of considering multiple modes of transportation. Considering the probability of cold chain interruption at each logistics transfer point as the cold chain interruption probability [13] is

(3) $$\begin{array}{c} d_{l}=D_{p}^{l}h_{1}^{l}{\left(1-h_{1}\right)}^{p-l}\text{.} \end{array}$$

Here, *D*_*p*_^*l*^ represents the probability of cold chain interruption at *l* transit points, *h*_1_^*l*^ represents the probability of cold chain interruption at 1 transit point, and *p* represents a total of *l* transit points.

Traffic congestion is also a key factor affecting the cold chain transportation of fresh products. This paper selects the k-nearest neighbor algorithm to predict the risk of traffic congestion. K-nearest neighbor algorithm is one of the simplest methods in data mining classification technology, which means that each sample can be represented by its nearest K neighbors. If most of the k-nearest samples in the feature space belong to a category, then a sample also belongs to that category and has the properties of samples in that category. K-nearest neighbor algorithm only determines the classification of the samples to be divided according to the category of the nearest one or several samples. When making a classification decision, it is only related to a very small number of adjacent samples. New data can be directly added to the data set without retraining. K-nearest neighbor algorithm is simple in theory, easy to implement, high in accuracy, and has a high tolerance to outliers and noise. Therefore, choosing a k-nearest neighbor algorithm to predict the risk of traffic congestion can effectively shorten the transportation time of cold chain logistics.

Through the collection and analysis of related data affecting traffic, build K-nearest neighbor prediction model state vector (*x*, *y*, *q*), according to the collected state vector data, the storage form is (*x*_*i*_, *y*_*i*_, *q*_*i*_), collected historical database should include a variety of possible factors of state vector and congestion index: for traffic congestion index prediction, first build state vector *Q*(*x*, *y*, *q*) according to the information that can be collected in advance.

Then, calculate the distance between the required state vector and the history vector (*x*_*i*_, *y*_*i*_, *q*_*i*_), search for the first K historical state vector with the shortest distance, and the predicted value is calculated using the TPI corresponding to the K state vectors. The value of the K-nearest neighbor algorithm is shown in Figure 3.

In the k-nearest neighbor algorithm, the distance is the judgment basis of the predicted state vector and the historical state vector. The smaller the distance is, the more similar the historical state vector is. This paper adopts the Euclidean distance calculation method. Euclidean distance is a commonly used definition of distance, which is the true distance between two points in m-dimensional space. The Euclidean distance in two and three dimensions is the distance between two points. Euclidean distance is simple, easy to operate, and widely used. The specific calculation formula is shown in the following formula:

(4) $$\begin{array}{c} dis\left(x_{i},y_{i},q_{i}\right)=\sqrt{{w_{i}\left(x_{i}-y_{i}\right)}^{2}}+\sqrt{{w_{i}\left(x_{i}-q_{i}\right)}^{2}}+\sqrt{{w_{i}\left(y_{i}-q_{i}\right)}^{2}}\text{.} \end{array}$$

The distance of change trend of congestion index refers to the difference between two time difference series, i.e., numerical difference and change trend difference. The calculation method used in this paper is the variance and correlation coefficient method, in which the greater the variance, the farther the distance between them, the smaller the correlation coefficient, the more uncorrelated, and the greater the distance between them. Assuming that the congestion index sequence of 3 h before the current moment is *F*_*i*_[*aF*_1_, *aF*_2_, ...*aF*_*m*_], the congestion index sequence of the same period in the historical library is a, and the number of elements of *f* and *a*_*i*_[*a*_*i*__1_, *a*_*i*__2_, ..., *a*_*i*__*m*_] is *m*, the change trend of the congestion index can be expressed as follows:

(5) $$\begin{array}{c} \alpha_{i}=\sqrt{\overset{n}{\underset{i=1}{\sum }}{\left(a_{i}-F_{i}\right)}^{2}}\text{.} \end{array}$$

Among them, *α*_*i*_ indicates the final trend of congestion index change.

## 4. Weight Calculation of Cold Chain Logistics Risk Factors Based on Analytic Hierarchy Process

According to the above-determined risk factors of fresh product export cold chain logistics transportation, in order to realize the decision-making and optimization of the transportation path, it is necessary to calculate the weight of these influencing factors to determine the key role of different influencing factors. The calculation of the risk factor weight of fresh product export cold chain logistics transportation is an extremely important aspect of risk control management. In enterprise risk management, when the risk evaluation result is a high risk, it is necessary to deal with and strictly control the risk, and the treatment means are relatively complex; When the risk assessment result is low risk, simple and effective risk control measures shall be taken or no risk control measures shall be taken according to the actual situation. The calculation of risk factor weight of fresh product export cold chain logistics transportation provides a theoretical basis for risk intelligent control of fresh product cold chain transportation. In the risk management of fresh product export cold chain logistics transportation, risk accidents are uncertain, the importance of risk factors is different, and the risk intelligent control methods are also different. In this paper, the analytic hierarchy process is used to quantitatively analyze the risk influencing factors of fresh product export cold chain logistics. Combined with the evaluation results, the intelligent control technology is used for risk control. Through the identification and monitoring of transportation risk factors through intelligent control technology, the risk of accident rate is reduced to the lowest; At the same time, it provides research ideas on expected identification, control, and evaluation for the risk management of fresh product export cold chain transportation.

The analytic hierarchy process (AHP) is a method combining qualitative analysis and quantitative analysis. According to the studied target problems, the influencing target factors are divided into different levels and then combined according to the relationship between the factors at different levels to build a multilevel framework model. Therefore, the problems are summarized as the ranking of advantages and disadvantages between the implementation scheme and the overall implementation goal and the measurement of relative importance. When using this method to build the calculation model, there are four steps: (1) establish the hierarchical structure model. 2. Build the judgment (pairwise comparison) matrix. 3. Hierarchical single ranking and its consistency test. 4. Hierarchical total ranking and its consistency test.

### 4.1. Establish Hierarchy Model

The hierarchical model uses concrete data structure to represent various entities and the relationships among them. Each node represents a record type, and the structure represents the relationships among entity types. The hierarchical model has a clear structure and simple connection between nodes. As long as we know the parent nodes of each node, we can know the whole model structure. Therefore, the establishment of the hierarchical model can effectively optimize the expected identification, control, and evaluation of fresh product export cold chain transportation risk management. The risk evaluation index system of fresh product export cold chain logistics transportation is divided into three hierarchical structures: target layer (layer a), criterion layer (layer B), and index layer (layer C).

### 4.2. Construction of Judgment Matrix

The value of the judgment matrix element is determined according to the comparison of two factors. The specific value method is expressed by santy's 1–9 scale method. It is more appropriate to compare less than 9 factors. Suppose there are *n* factors under layer a, and its judgment matrix can be expressed as follows:

(6) $$\begin{array}{c} W=\left[\begin{array}{c} \begin{array}{cccc} w_{11} & w_{12} & ... & w_{1n} \end{array}\\ \begin{array}{cccc} w_{21} & w_{22} & ... & w_{2n} \end{array}\\ ...\\ \begin{array}{cccc} w_{n1} & w_{n2} & ... & w_{nm} \end{array} \end{array}\right]\text{.} \end{array}$$

Set the judgment matrix as follows:

(7) $$\begin{array}{c} A={\left(w_{ij}\right)}_{n*m}\text{.} \end{array}$$

### 4.3. Level of Single Ranking and Its Consistency Inspection

#### 4.3.1. Level of Single Sorting

Hierarchical single ranking is to obtain the vector M, the feature vector W, and the maximum feature root *β*_max_ of the judgment matrix. The numerical size of the feature vector W element represents the weight arrangement of the lower layer relative to the upper layer. The specific calculation formula is as follows:

(8) $$\begin{array}{c} M={\left(\overset{n}{\underset{i=1}{\prod }}w_{ij}\right)}^{1/n}\left(i=1,2,\ldots ,n\right)\text{,} \end{array}$$

where *M* represents the normalized vector.

(9) $$\begin{array}{c} w_{ij}=\frac{M}{\underset{i,j=1}{\sum }M_{j}}\text{.} \end{array}$$

#### 4.3.2. Consistency Inspection

The reason for the consistency test is that things have diversity and human cognition has certain limitations. The specific inspection methods are as follows: define the consistency index: CI as follows:

(10) $$\begin{array}{c} CI=\frac{\beta_{\max}-n}{n-1}\text{,} \end{array}$$

where *β*_max_ represents the maximum eigenvalue of the judgment matrix; *n* value is the number of elements.

Hierarchical total rank consistency test, the hierarchical single rank consistency index of factor A in layer B layer is (*b*_1_, *b*_2_, ...*b*_*n*_), then the hierarchical total rank consistency ratio is

(11) $$\begin{array}{c} CR=\frac{\overset{n}{\underset{i=1}{\sum }}w_{ij}CI}{\overset{m}{\underset{j=1}{\sum }}RIw_{ij}}\text{.} \end{array}$$

Here, RI represents the relevance Indicator. When the CR is less than 0.1, the total ranking means that the consistency test is passed, otherwise the judgment matrix element with a high single ranking consistency ratio needs to be adjusted.

#### 4.3.3. Calculation of the Weight Result Value

Based on the above-given analysis, the weight of the risk factors of fresh products is calculated, and the calculation formula is

(12) $$\begin{array}{c} P_{i}=\overset{n}{\underset{i=1}{\sum }}w_{ij}CI\text{.} \end{array}$$

Among them, *P*_*i*_ indicates the weight results of the cold chain transportation of fresh products.

## 5. Cold Chain Logistics Route Decision Optimization Based on Genetic Algorithm

The traditional logistics transportation path problem is that without considering its own and external factors, the roads between distribution stations are directly connected. Logistics transportation vehicles start from the central warehouse, transport all distribution stations, and finally return to the central warehouse. All distribution stations are traversed only once. Therefore, this paper adopts a genetic algorithm [14] to realize the decision-making optimization of the cold chain logistics path for fresh product export. Genetic algorithm is famous for its fast search speed, high efficiency, simple structure, and easy control of parameters. So far, it has been studied and applied by the majority of researchers. Therefore, this paper uses a genetic algorithm to solve the logistics transportation path problem, so as to minimize the transportation path and improve the transportation efficiency. At the beginning of the calculation, a certain number of individuals are randomly initialized and the fitness value of each individual is calculated to generate the first generation (initial population). If the optimization criteria are not met, the calculation of a new generation is started, and individuals are selected according to the fitness value to produce the next generation. The parent generation will cross operate according to a certain probability to produce the offspring. All offspring mutate with a certain probability to form a new generation. Calculate the fitness value of the new progeny. This process is repeated until the optimization criteria are met to solve the optimal path problem.

The search object of the genetic algorithm is a group of solutions, not just a single solution. Firstly, all possible solutions of the problem are encoded according to certain rules to obtain the initialization individual, namely, chromosome. Then, according to certain rules and mechanisms, some chromosomes are selected to form the initial population; after the initial population is selected, the fitness of each chromosome in the population should be calculated, and the parent individuals used for heredity should be selected for replication according to the fitness; then select, cross and mutate the individuals according to the algorithm rules, and continuously generate new individuals through iteration to form a new population. The adaptability of these new individuals must be better than that of the previous generation, so as to ensure a stronger ability to adapt to the environment [15]; finally, when the population iterates to the specified algebra or the fitness of the population iterates to a certain algebra, there is no optimization trend. At this time, it can be judged that the individual here is the optimal individual of the population, and the optimal solution of the problem can be obtained by decoding it. The main implementation steps of the genetic algorithm are as follows:

Step 1: the result of solving the cold chain logistics path of fresh product export by the genetic algorithm is greatly affected by the quality of the initial solution, while the quality of the solution obtained by the randomly generated initial solution is usually poor. Based on various performance indicators and personal preferences, the decision-maker proposes to form an initial solution, that is, first divide the value range of each parameter to be optimized into groups and cells, and then randomly generate an initial individual in each cell. In this way, the initial individuals will be evenly distributed in the whole solution space and can ensure that the initial population contains rich patterns, which increases the possibility of converging to the global optimal solution. In this regard, this paper also proposes a decision-making method of fresh product export cold chain logistics path based on the time processing capacity index. This method first uses the randomly generated location sequence to sort each influencing risk factor and then randomly selects two risk indexes in each region. If the random value between 0 and 1 is less than 0.8, the best index is selected; If the random value between 0 and 1 is less than 0.8.
Step 2: encoding
Whether the coding is completed in the genetic algorithm is the key to successful optimization. The coding based on the process is the most widely used in traditional methods. Each process is represented by the corresponding serial number based on the coding chromosome. When the chromosome is scanned from left to right, the serial number *k* of the workpiece indicates the k-th machining of the workpiece. The advantage of this method is that the scheduling is feasible, deadlock is avoided, and the representation of solution space is complete. However, logistics path optimization requires not only determining the order of process selection but also selecting the best adapter for each process. Only using a process based coding method can not effectively deal with this problem. Aiming at this problem, an extended process based coding method is proposed. This method is divided into two different parts. The first is based on process coding, which can determine the order of the selection process. The other is based on location coding, which can set the corresponding reasonable location to all processes. The two coding methods are combined. The binary coding method is adopted to make the binary symbol set {0, 1} composed of binary symbols 0 and 1. A binary coding symbol string is an individual genotype, also known as a chromosome. If the value range of a parameter is [*U*_min_, *U*_max_], the code of individual *x* is *x*_*l*_*x*_*l*1_...*x*_1_*x*_0_.
Step 3: genetic operator
Genetic operation is basically the same as a traditional genetic algorithm, and its biggest feature is selective operation. The selection of genetic manipulation is generally divided into three parts. Firstly, the best and worst individuals in the current population are found according to the fitness value; secondly, if the fitness value of some individuals in the contemporary population is higher than that of the retained excellent individuals, the existing excellent individuals will be replaced by the contemporary excellent individuals; finally, the retained excellent individuals are used to eliminate the worst individuals in the next generation population. It is assumed that the population can be divided into m layers according to the level of noninferior solution. The smaller the index, the higher the noninferior solution level. For I individuals, if their noninferior solution level is *j* and individuals at the same noninferior solution level have the same fitness, it is called shared fitness. In order to make the optimization results evenly distributed in the target space, it is necessary to calculate the local crowding distance of individuals on each noninferior solution level. Based on the calculation of shared fitness and local crowding distance, parents were randomly selected. When the sharing fitness is different, individuals with higher sharing fitness can be selected. When the fitness is the same, select the individuals with a large local crowding distance. Repeat the above-given selection until offspring are formed.
Step 4: description of logistics path decision-making problem of fresh product export cold chain
This paper describes the optimization problem of cold chain logistics distribution as follows: when the geographical location of the distribution center and customers is known, according to the customer's demand for products and the arrangement of time, reasonably schedule the cold chain logistics transportation vehicles, and start from the distribution center to provide distribution services for customers in turn; Among them, the customer's demand is known, the customer's requirements for the arrival time window of goods are known, and the vehicle load and the maximum single driving distance are also known. It is required to formulate an efficient and reasonable vehicle distribution scheme on the premise of no repeated distribution, meeting the customer's needs, and meeting the constraints, so as to realize the optimization of the objective function. After the above-given analysis, the cost elements and expressions of each module of cold chain logistics have been established. This paper aims to minimize the total cost of comprehensive logistics distribution, and the final cold chain logistics path optimization model is expressed as follows:
  (13) $$\begin{array}{c} \min\;E=\min\;\left[\overset{n}{\underset{i=1}{\sum }}sign\left(k\right)+\overset{n}{\underset{j=1}{\sum }}w_{ij}p_{i}\right]\text{.} \end{array}$$

The number of refrigerated vehicles, that is, the number of final distribution routes, can be changed and adjusted according to the specific customer demand, so as to meet the demand without waste, as shown in the following formula:

(14) $$\begin{array}{c} T=\text{int}\left[\frac{\overset{n}{\underset{i=1}{\sum }}r_{i}}{T}\right]+1\text{.} \end{array}$$

Here, *T* represents the number of vehicles, *r*_*i*_ represents the demand of the customer ii, and *T* represents the maximum carrying capacity of the bicycle. The formula expresses the maximum carrying capacity of the customer with the total demand of the bicycle, and 1 is added as the number of vehicles in the final demand of cold chain logistics.

Fitness is used to evaluate the advantages and disadvantages of the determined distribution scheme. In the path optimization problem, a distribution scheme corresponds to a chromosome. The goal of this paper is that the smaller the distribution cost, the better. There is a negative correlation between fitness and target value. Therefore, the fitness value can be expressed by the reciprocal of chromosome objective function value.

Fit (i) indicates the fitness, and *C*_*t*_ represents the target function value of the *i* th chromosome. The relationship expression between the two is

(15) $$\begin{array}{c} Fit\left(t\right)=\frac{1}{C_{t}}\text{.} \end{array}$$

Among them, *C*_*t*_ represents the total cost of the distribution path in Article *i*, that is, the target function value of this paper, the smaller the total cost, the greater the fitness, the higher the feasibility, so the fitness function is feasible, so the design of the decision optimization method of the export cold chain logistics path of fresh products is completed.

## 6. Experimental Verification

### 6.1. Experimental Environment

In this experiment, Matlab is used and implemented in the running environment of the p4cpu program. The main frequency is 3.0 GHz and the memory is 512 MB. This case is divided into two parts. Firstly, the performance of the algorithm is tested and the test results are compared. The running parameters in the experiment include 200 population sizes, selection probability of 0.9, and maximum evolutionary algebra of 80. The area of cold chain transportation in this region is 15 km2. A well-known export company in China is selected to take its primary fresh product export cold chain logistics as the research object to optimize the logistics path. The specific arrival place of the fresh product in the cold chain logistics transportation is shown in Figure 4.

In Figure 4, circle 1 is the starting point of this transportation route. This transportation needs to be transported to circle 13 at the end point, passing through 11 parking spots. In this transportation, it should be driven according to the normal main roads in the map. In the experiment, by optimizing the constructed economic and environmental protection objective function, the values of the objective function are in the same quantitative range, that is, weighted average distribution. The unbalanced weight coefficient can be used to reflect different preference relationships in special cases. By defining the solution, each initial solution has at least one objective function value better than other objectives. The solution at the center of space is an unbiased optimal solution. Under the same conditions of concern, the objective function can choose the unbiased optimal solution as the optimal solution. Under the same conditions of concern, the objective function can choose the unbiased optimal solution as the optimal solution.

In the experiment, the methods of this paper, literature [7] and literature [8] are used to optimize the transportation route decision, and the experimental analysis is carried out with the accuracy of route decision, the time to reach the destination, and the error of route planning as the experimental indicators.

### 6.2. Experimental Results

#### 6.2.1. Impact Analysis of Traffic Route Decision

In the experiment, the method in this paper, the method in literature [7] and the method in literature [8] are used to optimize the transportation route decision. These three methods are used to make the initial route transportation decision. The effect of route decision is shown in Figure 5.

By analyzing the experimental results in Figure 5, it can be seen that the methods in this paper, literature [7] and literature [8] are used to optimize the transportation route decision. The routes after the initial route transportation decision are made by these three methods are different. Among them, the path decided by this method is the shortest and smoothest transportation path among the three methods. Compared with the path planned by the other two methods, there are more decisions of repeated sections, so it can be seen that this method is more feasible. This is because a genetic algorithm is used to improve the calculation effect of optimal cold chain logistics route decision function of new product export through encoding, decoding, crossover, and other operations, so as to improve the decision effect of traffic route.

#### 6.2.2. Analysis of Transportation Route Decision Accuracy

In the experiment, the method in this paper, the method in literature [7], and the method in literature [8] are used to optimize the transportation route decision. After using these three methods to make the initial route transportation decision, in order to reflect the data results of the method, the decision accuracy of the obtained route decision effect is quantified. The results are shown in Figure 6.

By analyzing the experimental results in Figure 6, it can be seen that there are some differences in the precision results of transportation route decision optimization by the methods in this paper, literature [7] and literature [8]. It can be seen that the precision of decision optimization using this method is about 90% of the average value, while the precision of decision optimization using the other two traditional methods is low and fluctuates. Therefore, it can be seen that the decision path using this method is more suitable and feasible. This is because the analytic hierarchy process (AHP) is used to take the transportation information of the cold chain logistics route of fresh product export as the value of the risk factor judgment matrix, so as to calculate the accurate index weight of the risk factor and improve the decision-making accuracy of the transportation route.

#### 6.2.3. Transporting Route Arrival Time Analysis

In the experiment, the transportation route decision optimization is carried out according to the methods in this paper, literature [7] and literature [8]. After using these three methods to make the decision of initial route transportation, the time when the transportation route of the three methods reaches the destination is analyzed. The results are shown in Table 2.

By analyzing the experimental results in Table 2, it can be seen that the method in this paper, the method in literature [7], and the method in literature [8] are used to optimize the transportation route decision. After using these three methods to make the initial route transportation decision, there is a certain difference in the time when the transportation route reaches the destination according to the three methods in the experiment. Among them, the shortest time is the method in this paper. Although the other two methods are within a reasonable range, they are longer than the method in this paper. This is because the transportation risk factor system of cold chain logistics for the export of new products considering the transportation risk is constructed, so as to optimize the customs clearance efficiency, vehicle stability, cold chain terminal, traffic congestion, and other factors of cold chain logistics and shorten the transportation time of cold chain logistics route. Therefore, it can be seen that the method in this paper is more feasible.

## 7. Conclusion

Based on the analysis of the shortcomings of the traditional cold chain logistics of fresh product export, the optimization method of the cold chain logistics route decision of fresh product export considering the transportation risk factors was proposed, which promoted the vehicle stability of the cold chain distribution link of fresh product export and reduced the traffic congestion. Through the method of risk quantification, the basic characteristics and classification of cold chain logistics are analyzed, and the transportation risk factor index system of cold chain logistics is constructed. The k-nearest neighbor algorithm is used to predict the risk of traffic congestion and extract the transportation risk factors of cold chain logistics, so as to shorten the transportation time. In order to reduce the error of path planning, ahp was used to construct a calculation model, and the index weight of risk factors was calculated by the risk factor matrix. A genetic algorithm is introduced to construct the optimal decision function of the cold chain logistics route of new product export through encoding, decoding, crossover, and other operations and optimize the decision of the cold chain logistics route of fresh product export. Experimental results show that the method proposed in this paper can improve the effect of cold chain logistics route decision, the accuracy of decision optimization is about 90%, and the time to reach the destination is short, reduce the transport time, with a certain transport efficiency.

## Figures and Tables

**Figure 1:** General process diagram of cold chain logistics.

**Figure 2:** Risk factor index system of cold chain logistics transportation for fresh product export.

**Figure 3:** Schematic diagram of k-nearest neighbor algorithm.

**Figure 4:** Schematic diagram of export cold chain transportation path of sample fresh products.

**Figure 5:** Analysis on the effect of different decision-making methods on transportation route decision-making.

**Figure 6:** Analysis of decision accuracy of transportation route with different decision-making methods.

**Table 1:** Classification of cold chain logistics storage environment.

Storage environment	Temperature (°C)	Product
Ultralow temperature	≤−30	Tuna, reagents, vaccines, etc
Freeze	−23–18	Frozen meat, frozen food
Keep in cold storage	0–8	Cold fresh meat, fresh milk, fruits and vegetables, etc

**Table 2:** Time analysis of transportation routes reaching the destination by different decision-making methods (min).

Number of iterations	Paper method	Literature [7] methods	Literature [8] methods
10	30.21	39.41	38.52
20	31.20	40.12	41.20
30	30.85	41.20	41.35
40	30.41	42.13	41.69
50	32.10	42.96	42.10
60	32.14	43.10	42.13
70	31.89	43.21	43.12
80	32.41	44.21	44.15
90	30.41	45.21	45.31
100	31.45	45.32	45.21

## Data Availability

The dataset can be accessed from the corresponding author upon request.
